# Clinical Value of the Prognostic Nutrition Index in the Assessment of Prognosis in Critically Ill Patients with Stroke: A Retrospective Analysis

**DOI:** 10.1155/2022/4889920

**Published:** 2022-05-09

**Authors:** Yang Liu, Xiaobin Yang, Sultan Kadasah, Chaosheng Peng

**Affiliations:** ^1^Department of Health Medicine, The Sixth Medical Center of PLA General Hospital, Beijing, China; ^2^Day Clinic Area, The Sixth Medical Center of PLA General Hospital, Beijing, China; ^3^Department of Biology, Faculty of Science, University of Bisha, Saudi Arabia

## Abstract

**Purpose:**

The purpose of study was to evaluate the association between prognostic nutritional index (PNI) and all-cause mortality of critically ill patients with stroke.

**Methods:**

Clinical data derived from Multiparameter Intelligent Monitoring in Intensive Care were analyzed. The primary endpoint was 30-day all-cause mortality; secondary endpoints were 90-day mortality and one-year cause mortality. The potential prognostic roles of PNI were analyzed by Cox proportional hazard models. The independent prognostic roles of PNI in the cases were analyzed by smooth curve fitting.

**Results:**

Concerning 30-day mortality, the HR (95% CI) for a high PNI (≥39.7) was 0.700 (0.544, 0.900; *P* = 0.00539), compared to a low PNI (<39.7). After adjusting for multiple confounders, the HR (95% CI) for a high PNI (≥39.7) was 0.732 (0.547, 0.978; *P* = 0.03514), compared to a low PNI (<39.7). Regarding 90-day and one-year mortality, a similar trend was observed. In addition, a nonlinear association between PNI and 30-day mortality was found. Using recursive algorithm and two-piecewise linear regression model, inflection point (IP) was calculated, which was 49.4. On the right side of the IP, there was a positive relationship between PNI and 30-day mortality, and the effect size, 95% CI, and *P* value were 1.04 (1.01, 1.07), *P* = 0.0429, respectively. On the left of the IP, the effect size, 95% CI, and *P* value were 0.97 (0.96, 0.99) and 0.0011, respectively.

**Conclusions:**

The PNI was an independent predicting factor of 30-day, 90-day, and 1-year mortality of the critically ill patients with stroke. In addition, there was a U-shaped relationship between PNI and all-cause mortality of stroke patients. PNI was a risk factor for the outcome of stroke when PNI was >49.4, while PNI was a protective factor for outcome of stroke when PNI was <49.4.

## 1. Introduction

Stroke ranks the first among the fatal diseases in China [1]. It is also the main illness causing disability in Chinese adults [2], which is featured by high incidence, high mortality, and high disability rates. It is observed that cases with the first stroke may have another stroke or repeated stroke after a period of rehabilitation in hospital [3]. Among the cases in intensive care unit (ICU), those with critical stroke account for a large proportion [3]. There is a lack of effective treatment for stoke, causing great loss and burden to the family and society. Thus, it is necessary to find a biomarker to predict the prognosis of stroke cases in an early stage [4].

Inflammation is involved in the pathology and outcomes of acute stroke [5, 6]. Several studies showed that inflammatory biomarkers, neutrophil-to-lymphocyte ratio [7], platelet-to-lymphocyte ratio [8], red blood cell distribution width-to-albumin ratio [9], and red blood cell distribution width [10] could be used to predict the outcome of cases with stroke. However, these biomarkers are relatively homogeneous and not comprehensive. Prognostic nutritional index (PNI) is a new prognostic score which is calculated from serum albumin level and total lymphocyte count. Previous studies indicated that a higher level of lymphocytes could upregulate the anti-inflammatory cytokine interleukin (IL)-10 and suppress inflammatory cytokines including tumor necrosis factor (TNF)-*α* and IL-6, which can play an anti-inflammatory effect [10]. In addition, clinical evidence shows that lower lymphocyte count is associated with poor early neurological function improvement and poor long-term functional prognosis [11]. Likewise, albumin serves as a neuroprotective factor given the anti-inflammatory, antioxidant, and antiapoptotic properties [12]. It was illustrated that a reduced Albumin level was closely linked to worse outcomes of cases with stroke. Therefore, PNI is a combination of lymphocytes and albumin which can simultaneously evaluate the overall inflammation and nutritional conditions of the patients with stroke.

Recent evidence showed that PNI was closely associated with clinical outcomes of cancer [13, 14] and sepsis [15, 16]. However, the prognostic role of PNI in the cases with stroke is still unclear. Therefore, this study is aimed at exploring associations between PNI and outcomes of patients with stroke.

## 2. Methods

### 2.1. Data Source

The study was carried out based on the Strengthening the Reporting of Observational Studies in Epidemiology (STROBE) statement [17]. Data were obtained from the Multiparameter Intelligent Monitoring in Intensive Care III (MIMIC-III) version 1.4, containing vital signs, medications, demographic information, and other related data of the cases admitted to intensive care unit from 2001 to 2012 in the Beth Israel Deaconess Medical Center (BIDMC), Boston. The protocol was approved by Massachusetts Institute of Technology (MIT) and the Institutional Review Boards.

Of the cases recorded in the MIMIC-III database, stroke cases (>16 years old) upon the first admission with hospitalization period over one day were chosen. Exclusion criteria: (a) acute infection; (b) malignancy, critical hepatic illness, and kidney diseases.

### 2.2. Study Variables and Outcomes

Laboratory features, demographic data (e.g., race, gender, and age), comorbidities, vital signs, and scoring systems of the cases were collected. Laboratory measurements included albumin, white blood cell (WBC) count, platelet count, anion gap, chloride, blood urea nitrogen (BUN), and serum creatine in the first 24 hours. Comorbidities included coronary heart disease (CHD), atrial fibrillation (AF), and heart failure (HF). Vital signs monitored in the first 24 hours included heart rate, oxygen saturation (SPO_2_), diastolic blood pressure (DBP), systolic blood pressure (SBP), and mean arterial pressure (MAP); systemic inflammatory response syndrome (SIRS) score, sequential organ failure assessment score(SOFA), and simplified acute physiology score (SAPS II) were also included. PNI was calculated as serum albumin concentration (g/l) + 0.005 × total lymphocyte count. After admission, the cases were followed up until death.

The clinical primary endpoint was 30-day all-cause mortality. The secondary endpoints were 90-day mortality and one-year all-cause mortality.

### 2.3. Statistical Analysis

To investigate whether PNI was related to the outcome of stroke cases, three main steps were taken for statistical analysis. Firstly, the optimal cutoff value for PNI was determined using the receiver-operating characteristics (ROC) curve. Categorical data were described as frequency or percentage and continuous results as mean ± standard deviation (SD). Continuous variables and categoric variables were compared between subgroups of PNI using *χ*^2^ and Kruskal-Wallis *H* tests, respectively. In the second step, cox proportional hazards model was used to assess the association between PNI with the mortality of critically ill patients with stoke. Results were presented as hazard ratios (HRs) with 95% confidence intervals (CIs). And we constructed three statistical models, including model I, model II, and model III. In model I, no covariate was adjusted; in model II, only ethnicity, sex, and age were adjusted; in model III, ethnicity, sex, age, DBP, SBP, heart rate, SPO2, respiratory rate, temperature, SOFA, chloride, and AF were adjusted. In the third step, smooth curve fitting was used to analyze the independent predicting role of PNI in the mortality of the stroke cases.

Two-sided *P* value < 0.05 was considered statistically significant. Statistical Product and Service Solutions (SPSS) software (version 27.0) was used to conduct all statistical analyses of this study.

## 3. Results

### 3.1. Subject Characteristics

In our study, 958 stroke cases were included. The baseline demographic, laboratory, and clinical features of the participants are listed in Table 1. The eligible participants included 516 women and 420 men with a mean age of 67.46 ± 15.37 years, and the mean PNI was 43.08 ± 24.37. It was demonstrated that the proportions of cases with HF or AF, 30-day, 90-day, and one-year mortality were increased in the low PNI group (PNI < 39.7). The SBP, DBP, MAP, temperature, and SpO_2_ were decreased (*P* < 0.05). Moreover, organ function was also assessed in the two groups using the laboratory indices, and the results showed that hepatic and renal function of patients in the low PNI group was worse than that in the high PNI group.

### 3.2. Association of PNI with 90-Day, 30-Day Mortality, and One-Year Mortality of Cases with Stroke

In our study, three models were constructed to assess independent prognostic roles of PNI in stroke cases after adjustment of other possible confounders. 95% CI and effect sizes (HR) are listed in Table 2. Concerning 30-day mortality, the HR (95% CI) for the high PNI (≥39.7) was 0.700 (0.544, 0.900; *P* = 0.00539), compared to the low PNI (<39.7). In model 2, ethnicity, sex, and age were adjusted, and the HR (95% CI) for the high PNI (≥39.7) was 0.701 (0.545, 0.902; *P* = 0.00579), compared to the low PNI (<39.7). In model 3, a variety of confounders (race, sex, age, heart rate, DBP, SBP, temperature, respiratory rate, SPO2, SOFA, chloride, and AF) were adjusted, and the HR (95% CI) for the high PNI (≥39.7) was 0.732 (0.547, 0.978; *P* = 0.03514), compared to the low PNI (<39.7).

Regarding 90-day mortality, a similar trend was observed. In model I, the HR (95% CI) for the high PNI (≥39.7) was 0.625 (0.498, 0.786; *P* = 0.00006), compared to the low PNI (<39.7). In model 2, ethnicity, sex, and age were adjusted, and the HR (95% CI) for the high PNI (≥39.7) was 0.628 (0.499, 0.789; *P* = 0.00007), compared to the low PNI (<39.7). In model 3, a variety of confounders (race, sex, age, heart rate, DBP, SBP, temperature, respiratory rate, SPO2, SOFA, chloride, and AF) were adjusted, and the HR (95% CI) for the high PNI (≥39.7) was 0.704 (0.541, 0.916; *P* = 0.00886), compared to the low PNI (<39.7). For one-year mortality, a similar trend was observed.

### 3.3. Nonlinear Relationship

Using the generalized additive model, nonlinear relationship of PNI with the 30-day mortality was analyzed (Figure 1). The two-piecewise LRM (linear regression model) and LRM were analyzed, and the *P* value was 0.012 revealed by the log-likelihood ratio test, demonstrating that the two-piecewise LRM fit the model. Using two-piecewise LRM and recursive algorithm, the IP (inflection point) was calculated, which was 49.4 (Table 3). On the right side of the IP, there was a positive association of PNI with 30-day mortality, and the effect size, 95% CI, and *P* value were 1.04 (1.00, 1.07), and 0.0429, respectively. On the left side of the IP, the effect size, 95% CI, and *P* value were 0.97 (0.96, 0.99) and 0.0011, respectively. U-shape between PNI and 30-day mortality threshold of 49.4 was found. Taken together, it was demonstrated that PNI had a threshold effect on the 30-day mortality.

## 4. Discussion

In our mind, this is the first comprehensive study to explore the correlations between PNI and the short-term and long-term mortality of cases with acute stroke. In our study, it was found that higher FAR was closely related to the increased short-term and long-term mortality of all causes in those who suffered from acute stroke. The results of nonlinear relationship analysis in the study suggested U-shape between PNI and the 30-day mortality, with a threshold of 49.4.

Systemic inflammation is critical in stroke development and progression [18, 19]. Indeed, in stroke, disease progression is associated with nonspecific and subclinical inflammatory processes. However, immunologic mechanism is also reported to be involved in stroke, although it remains be further investigated [20]. Monocytes, neutrophils, leukocytes, and platelets are dysregulated [21], which are related to inflammatory cascade. They regulate a variety of endocrine and paracrine signals, recruit additional cells, elicit generation and release of proinflammatory factors, and promote the expression of factors or receptors that are receptive to additional inflammatory signals possibly involved in disease progression [22]. Systemic inflammation was featured by alteration of circulatory platelets and white blood cells; thus, blood cell-based scores/ratios were calculated. Therefore, the prognostic roles of subclinical inflammation are further investigated.

Albumin can exert a neuroprotective effect and facilitate tissue recovery after brain ischemia due to the long acting period and half-life [23]. Some research [23–25] implied that a low level of albumin was related to stroke development and worse outcomes. It has been widely proved that albumin treatment could obviously decrease the infarction size and edema in brain.

Leukocytosis is associated with atherosclerotic disease severity, which is also reported to be related to unstable plaques and elicits acute thrombotic events [26]. Endothelial responses are featured by elevated expressions of proinflammatory cytokines and cellular adhesion molecules in atherosclerotic lesions, which promote activation and accumulation of leukocytes [27]. An inflammatory reaction is elicited by tissue hypoxia in the brain parenchyma of cases with acute ischemic stroke [28]. During the first 3 days after onset, peripheral vascular leukocytes are recruited, which elicit cerebral ischemic injury via several pathways. First, leukocyte adhesion to endothelia reduces microvasculature permeability and decreases erythrocyte flow, and brain no-reflow and further brain injury are hence caused. Collagenase, gelatinase, ROS, and proteases are secreted by activated leukocytes on the surface of damaged brain tissues and blood vessels. Second, activated phospholipase in leukocytes promotes secretion of active substances, e.g., prostaglandins, eicosanoids, platelet activating factors, and leukotrienes, which induce vasoconstriction and prolong platelet aggregation [29]. At last, some immune modulators and proinflammatory cytokines are secreted by infiltrated leukocytes in the penumbra zone around the infarct center, which may damage more neurons [30].

As a combined biomarker of lymphocytes and albumin, PNI is simple, efficient, and easy to obtain [15]. In addition, PNI can reflect the severity of inflammation and the nutritional status of the disease at the same time. Based on our results, the novel biomarker of PNI can be used to significantly predict stroke prognosis via lymphocyte and albumin levels.

Our research is mainly advantaged by in-depth analysis and large sample size, which is the first cohort study which assesses prognostic roles of PNI in acute stroke cases admitted to ICU. Nevertheless, there are also some limitations. First, this study is a retrospective cohort study, and some biases cannot be avoided. Although the association between PNI and mortality has been observed, this does not prove causality of that relation. Experimental as well as clinical observations are needed to further explore the mechanisms through which PNI may affect clinical outcome after stroke. Second, because of the limitation of the database itself, some variables cannot be collected, which affects the accuracy of the model, including proinflammatory factors and C-reactive protein. Third, only PNI in the first day of admission was analyzed, and the relationship between PNI over time and prognosis remains to be explored. Baseline assessment only was performed, which may lead to misclassification bias.

## 5. Conclusions

The PNI was an independent predicting factor of 30-day, 90-day, and 1-year mortality of the critically ill patients with stroke. In addition, there was a U-shaped relationship between PNI and all-cause mortality of stroke patients. PNI was a risk factor for the outcome of stroke when PNI was >49.4, while PNI was a protective factor for outcome of stroke when PNI was <49.4.

## Figures and Tables

**Figure 1:** The nonlinear relationship between PNI and all-cause mortality in patients with stroke revealed by the generalized additive model. (a) 30-day all-cause mortality; (b) 90-day all-cause mortality; and (c) one-year all-cause mortality.

**Table 1:** Baseline characteristics of the study population.

Characteristics	All	PNI		*P* value
		<39.7	≥39.7	
Number of patients	940	361	719	
Age, years	67.46 ± 15.37	68.26 ± 14.88	66.97 ± 15.66	0.270
Sex, *n* (%)				0.185
Male	424 (45.11)	153 (42.38)	271 (46.80)	
Female	516 (54.89)	208 (57.62)	308 (53.20)	
Ethnicity, *n* (%)				0.832
White	669 (71.17)	261 (72.30)	408 (70.47)	
Black	82 (8.72)	30 (8.31)	52 (8.98)	
Other	189 (20.11)	70 (19.39)	119 (20.55)	
Vital signs				
SBP, mmHg	127.12 ± 18.12	121.47 ± 17.64	130.63 ± 17.53	<0.001
DBP, mmHg	63.57 ± 11.36	61.22 ± 10.79	65.04 ± 11.47	<0.001
MAP, mmHg	82.17 ± 11.74	79.20 ± 11.39	84.01 ± 11.59	<0.001
Heart rate, beats/min	83.26 ± 16.39	86.69 ± 17.06	81.12 ± 15.61	<0.001
Temperature, °C	36.94 ± 0.69	36.92 ± 0.74	36.95 ± 0.66	<0.001
SpO2, %	97.60 ± 2.23	97.58 ± 2.45	97.60 ± 2.09	<0.001
Respiratory rate, t/min	19.05 ± 4.02	20.21 ± 4.56	18.32 ± 3.45	<0.001
Comorbidities				
Heart failure, *n* (%)	106 (11.28)	60 (16.62)	46 (7.94)	<0.001
Atrial fibrillation	282 (30.00)	128 (35.46)	154 (26.60)	0.004
CHD, *n* (%)	163 (17.34)	61 (16.90)	102 (17.62)	0.777
Laboratory parameters				
PNI	43.08 ± 24.37	33.25 ± 5.28	49.21 ± 29.15	<0.001
Albumin, g/dl	3.51 ± 0.69	2.87 ± 0.52	3.90 ± 0.45	<0.001
WBC, 10^9^/l	14.11 ± 8.98	14.11 ± 8.98	14.90 ± 16.24	0.284
Platelet, 10^9^/l	236.95 ± 122.21	217.00 ± 143.43	249.39 ± 105.10	<0.001
Lymphocyte, %	13.66 ± 11.03	10.18 ± 10.50	15.83 ± 10.80	<0.001
Creatinine, mg/dl	1.62 ± 2.05	1.88 ± 1.68	1.46 ± 2.24	<0.001
BUN, mg/dl	29.03 ± 23.39	37.29 ± 29.03	23.86 ± 17.12	<0.001
Serum chloride, mg/dl	107.54 ± 6.85	108.54 ± 7.20	106.92 ± 6.55	0.005
Anion gap, mg/dl	17.09 ± 4.28	17.22 ± 4.81	17.01 ± 3.92	0.869
Scoring systems				
SAPSII score	2.81 ± 1.01	45.84 ± 14.46	36.73 ± 13.41	<0.001
SOFA score	4.73 ± 3.29	6.20 ± 3.77	3.81 ± 2.56	<0.001
SIRS score	2.81 ± 1.01	3.01 ± 0.93	2.69 ± 1.04	<0.001
Clinical outcomes, *n* (%)				
30-day mortality	244 (25.96)	114 (31.58)	130 (22.45)	<0.001
90-day mortality	244 (25.96)	144 (39.89)	151 (26.08)	<0.001
One-year mortality	295 (31.38)	170 (47.09)	179 (30.92)	<0.001
Length of stay in ICU	6.84 ± 8.16	8.68 ± 8.90	5.69 ± 7.45	<0.001
Length of stay in hospital	13.32 ± 13.59	16.13 ± 15.05	11.56 ± 12.29	<0.001

Abbreviations: PNI: prognostic nutritional index; SBP: systolic blood pressure; DBP: diastolic blood pressure; MAP: mean arterial pressure; SAPSII: simplified acute physiology score II; SOFA: sequential organ failure assessment; ICU: intensive care unit; WBC: white blood cell; CHD: coronary heart disease; BUN: blood urea nitrogen.

**Table 2:** HR (95% CIs) for all-cause mortality across groups of PNI.

PNI	Model 1^a^		Model 2^b^		Model 3^c^	
	HR (95% CIs)	*P* value	HR (95% CIs)	*P* value	HR (95% CIs)	*P* value
30-day all-cause mortality						
<39.7	1.0		1.0		1.0	
≥39.7	0.700 (0.544, 0.900)	0.00539	0.701 (0.545, 0.902)	0.00579	0.732 (0.547, 0.978)	0.03514
90-day all-cause mortality						
<39.7	1.0		1.0		1.0	
≥39.7	0.625 (0.498, 0.786)	0.00006	0.628 (0.499, 0.789)	0.00007	0.704 (0.541, 0.916)	0.00886
One-year all-cause mortality						
<39.7	1.0		1.0		1.0	
≥39.7	0.610 (0.494, 0.752)	<0.0001	0.614 (0.498, 0.758)	<0.0001	0.725 (0.569, 0.924)	0.00939

Notes: models 1, 2, and 3 were derived from Cox proportional hazards regression models. (a) Model 1 covariates were adjusted for nothing; (b) model 2 covariates were adjusted for age, sex, and race; (c) model 3 covariates were adjusted for age, sex, race, heart rate, SBP, DBP, respiratory rate, temperature, SPO2, SOFA, chloride, and AF.

**Table 3:** Nonlinearity addressing by weighted two-piecewise linear model.

Outcome	30-day mortality HR (95% CIs) *P* value
Linear regression model	0.99 (0.97, 1.00) 0.0370
Two-piecewise linear regression model	
Inflection point	49.4
<49.4	0.97 (0.96, 0.99) 0.0011
≥49.4	1.04 (1.01, 1.07) 0.0529
Log likelihood ratio test	0.012

## Data Availability

All data included in this study are available upon request by contact with the corresponding author (Chaosheng Peng MD, E-mail: mailto:pengchaosheng@mail.chzu.edu.cn).
